This article has been retracted.

# DA Negatively Regulates IGF-I Actions Implicated in Cognitive Function via Interaction of PSD95 and nNOS in Minimal Hepatic Encephalopathy

**DOI:** 10.3389/fncel.2017.00258

**Published:** 2017-09-06

**Authors:** Saidan Ding, Weishan Zhuge, Xuebao Wang, Jianjing Yang, Yuanshao Lin, Chengde Wang, Jiangnan Hu, Qichuan Zhuge

**Affiliations:** ^1^Zhejiang Provincial Key Laboratory of Aging and Neurological Disease Research, Department of Surgery Laboratory, First Affiliated Hospital of Wenzhou Medical University Wenzhou, China; ^2^Gastrointestinal Surgery, First Affiliated Hospital of Wenzhou Medical University Wenzhou, China; ^3^Analytical and Testing Center, Wenzhou Medical University Wenzhou, China; ^4^Neurosurgery Department, First Affiliated Hospital of Wenzhou Medical University Wenzhou, China; ^5^Neurology Department, First Affiliated Hospital of Wenzhou Medical University Wenzhou, China

**Keywords:** minimal hepatic encephalopathy, dopamine, insulin-like growth factor I, ERK1/2/RSK pathway, PSD95–nNOS interaction

## Abstract

Insulin-like growth factor I (IGF-I) has been positively correlated with cognitive ability. Cognitive decline in minimal hepatic encephalopathy (MHE) was shown to be induced by elevated intracranial dopamine (DA). The beneficial effect of IGF-I signaling in MHE remains unknown. In this study, we found that IGF-I content was reduced in MHE rats and that IGF-I administration mitigated cognitive decline of MHE rats. A protective effect of IGF-I on the DA-induced interaction between postsynaptic density protein 95 (PSD95) and neuronal nitric oxide synthase (nNOS) was found in neurons. Ribosomal S6 protein kinase (RSK) phosphorylated nNOS in response to IGF-I by recruiting extracellular signal-regulated kinase (ERK1/2). In turn, DA inactivated the ERK1/2/RSK pathway and stimulated the PSD95–nNOS interaction by downregulating IGF-I. Inhibition of the interaction between PSD95 and nNOS ameliorated DA-induced memory impairment. As DA induced deficits in the ERK1/2/RSK pathway and the interaction between PSD95 and nNOS in MHE brains, IGF-I administration exerted a protective effect via interruption of the interaction between PSD95 and nNOS. These results suggest that IGF-I antagonizes DA-induced cognitive loss by disrupting PSD95–nNOS interactions in MHE.

## Introduction

Minimal hepatic encephalopathy (MHE) is indicated by mild disruption in psychomotor skills, cognition, or bimanual and visuo-motor coordination, which can be demonstrated using psychometric tests (Wein et al., 2004; Montoliu et al., 2007). However, if the diagnosis is made early in the process of the disease, these characteristics are reversible (Blei et al., 2001). Patients in the early stages of cirrhosis disease often manifest MHE. MHE can eventually develop into clinical HE and this leads to more serious alterations in intellectual functions, consciousness and coordination, which, in the most severe cases, can progress to coma and even death (Romero-Gómez et al., 2001). The pathogenesis of MHE and therapeutic drugs remains to be investigated.

Elevation of dopamine (DA) levels has been reported to be associated with neurological and psychiatric disorders (Beaulieu and Gainetdinov, 2011; Ungless and Grace, 2012). In our previous study, cognitive impairment in MHE was confirmed to be attributed to elevation of intracranial DA. However, the mechanism underlying the effects of DA on pathogenesis of MHE remains unclear. The toxic actions of DA appear to involve several distinct mechanisms including autoxidation, followed by oxidative stress, and D1 receptor activation (Chen et al., 2004). Importantly, DA released by midbrain dopaminergic neurons in both the striatum and the substantia nigra (Cheramy et al., 1981) controls GABA release through activation of D1 receptors located at the somato-dendrites and terminals of striato-nigral medium spiny neurons (Acosta-García et al., 2009). In addition, we have reported that DA influenced astrocyte function (Ding et al., 2014b,c, 2016). Therefore, it is imperative to elucidate the underlying pathogenesis of MHE as well as the appropriate therapeutic drug. Our several previous studies have indicated that intracranial DA overload is associated with cognitive impairment through more than one signaling pathway in MHE rats (Ding et al., 2013, 2014a,b,c). There is a pressing need to better understand this pathogenesis and find an effective therapeutic drug for DA-induced MHE disease.

Recently, it was shown that insulin-like growth factor I (IGF-I) is a neuroprotective factor that is involved in brain functions, including regulation of neuronal survival, neurogenesis, learning and memory, cognitive function and lifespan (Sonntag et al., 2005; Aleman and Torres-Alemán, 2009; Aksu et al., 2012; Ozdemir et al., 2012). IGF-I can pass through the blood-brain barrier (Reinhardt and Bondy, 1994) and plays important roles in neurocognitive ability in adults (Aksu et al., 2012; Ozdemir et al., 2012). In addition, it has been suggested that reduction of IGF-I levels is important in the process of age-related cognitive loss in humans (Aleman and Torres-Alemán, 2009). Recently, a meta-analysis indicated that there was a positive correlation between low levels of circulating IGF-I and cognitive impairment in the elderly who are healthy (Arwert et al., 2005). Furthermore, impaired IGF-I signaling influences the neurodegeneration cascade and leads to cognitive deficits and dementia-associated behaviors (de la Monte and Wands, 2005). Thus, impairment of IGF-I signaling appears to be a critical factor in development of cognitive deterioration in the brain. The question of whether cognitive disturbances can be prevented with IGF-I replacement therapy in MHE must be studied.

Postsynaptic density protein 95 (PSD95), which is also called synapse-associated protein-90 (SAP90), is a scaffolding protein that binds to neuronal nitric oxide synthase (nNOS) molecules at excitatory synapses. It then assembles them into a macromolecular signaling complex (Fukaya and Watanabe, 2000). Activated nNOS then catalyzes overproduction of highly reactive nitric oxide (NO) and induces NO toxicity (Dawson et al., 1993). Activation of nNOS depends on its association with PSD95 (Hu et al., 2013). Disrupting the interaction between PSD95 and nNOS can inhibit downstream nNOS signaling without blocking synaptic activity (Lai et al., 2011). nNOS enzyme activity, which is activated by binding to PSD95, leads to neurotoxicity that may be involved in cognitive function (Fukaya and Watanabe, 2000; Hu et al., 2013). Therefore, the nNOS–PSD95 interaction seems to play a key role in cognitive loss in MHE.

Therefore, it is of practical and theoretical interest to assess whether systemically administered IGF-I stimulates phosphorylation of nNOS and disrupts the nNOS–PSD95 interaction to preserve cognitive function in MHE. The goal of our study was to test the following hypotheses: (1) IGF-I can trigger disruption of the nNOS–PSD95 interaction to mediate memory function; (2) IGF-I can trigger phosphorylation of nNOS to disrupt the nNOS–PSD95 interaction via an extracellular signal-regulated kinase 1/2/ribosomal S6 protein kinase (ERK1/2/RSK) pathway; (3) DA blocks disruption of the nNOS–PSD95 interaction in MHE rats, which is IGF-I-mediated; and (4) Systemically administered IGF-I can enhance cognitive function through the ERK1/2/RSK/nNOS axis in MHE rats.

## Materials and Methods

### MHE Models and Treatments

Sprague-Dawley rats from the Experimental Animal Center of the Chinese Academy of Sciences in Shanghai, weighing 220–250 g, were used. Rats were maintained under a controlled temperature (24 ± 1°C) and controlled light (12 h light starting at 07:00 am) conditions. All experiments were carried out in accordance with the guidelines laid down by the Ethics Committees of the Affiliated Hospital of Wenzhou Medical University regarding the care and use of animals for experimental procedures (Albrecht et al., 2000).

Before experimenting, all animals underwent two behavioral tests: the Y-maze and the water-finding tasks. Normal values for these behavioral tests were acquired. The rats were randomly divided into two groups: a control group (*n* = 10) and a thioacetamid (TAA) group (*n* = 45). Liver cirrhosis was induced by intraperitoneal injection of TAA (200 mg/kg in normal saline, Sigma-Aldrich) twice per week for 8 weeks. TAA-treated rats that had symptoms were diagnosed with hepatic encephalopathy (HE). The symptoms of HE consisted of development of lethargy, decreased motor activity and an eventual progression to coma. TAA-treated rats that had no HE symptoms were then subjected to behavioral tests again to confirm that they had MHE or not. If TAA-treated rats met one of the following criteria, they were placed in the MHE group: (a) Y-maze score lower than the mean ± 1.96·SD; (b) water-finding tasks score higher than the mean ± 1.96·SD. Thirty-nine TAA-treated rats were placed in the MHE group. MHE rats were treated subcutaneously with IGF-I at a dose of 120 μg/kg per day, which was administered every 3 weeks for 3 months. They were also subjected to Y-maze and water-finding tasks tests or were treated with an intracerebroventricular (ICV) administration of IC87201 (100 nmol/10 μl infusion). Then the rats were subjected to the Y-maze and the water-finding tasks.

### DA-Treated Rat Models and Treatments

The remaining rats (*n* = 40) were also randomly divided into two groups: a DA-treated group (*n* = 30) and a control group (*n* = 10). Rats were anesthetized with an intraperitoneal injection of 10% chloralhydrate (0.4 g/kg). The rats were then placed on a stereotaxic apparatus. An injection (ICV) of DA hydrochloride (10 μg/3 μl in saline) was stereotaxically injected in the left lateral ventricle of rats three times at 7-day intervals (anterior–posterior, 0.3 mm; lateral, 1.0 mm; horizontal, 3.0 mm from the bregma; *n* = 30). Rats were tested in the Y-maze test and water-finding task at 24 h after the injection. DA-treated rats were subcutaneously injected with IGF-I at a dose of 120 μg/kg per day administered every 3 weeks for 3 months. Alternatively, they were treated with an ICV administration of IC87201 (100 nmol/10 μl infusion). Then the rats were subjected to the Y-maze test and water-finding task. They were subsequently sacrificed to collect the liver tissues, blood and brain tissues.

### Y-maze Test

The apparatus for the Y-maze task was made of gray plastic and each arm was 40 cm long, 12 cm high, 3 cm wide at the bottom and 10 cm wide at the top. The three arms were joined at an angle of 120°. The rats were placed individually at the end of an arm. The rats were permitted to move around the maze unrestricted for 8 min. The total arm entries and spontaneous alternation percentage (SA%) were recorded. We defined SA% as the ratio of the arm choices that differed from the previous two choices (“successful choices”) over the total choices during the run. This was considered as “total entries minus two” because the first two entries could not be evaluated. If a rat made 10 entries, for example, 1-2-3-2-3-1-2-3-2-1, there were five successful choices in eight total choices (10 entries minus 2).

### Water-Finding Task

We conducted water-finding task to assess the retention of spatial attention of the rats or latent learning (Mamiya et al., 1998; Kawasumi et al., 2004). The testing apparatus was composed of a gray plastic rectangular open field (50 × 30 cm, with a black 10 cm^2^ grid) with a 15 cm wall. A cubic alcove (10 × 10 × 10 cm) was attached to the center of the longer wall. A drinking tube was inserted through a hole at the center of the alcove ceiling. The tip of the tube was placed at 5 cm from the floor for training or at 7 cm for the trial. First we placed the rat in the near-right corner of the apparatus and it was allowed to walk around unrestricted for 3 min. Rats were omitted from the study when they did not find the tube within the 3-min exploration. Rats were deprived of water for 24 h after the training session. Rats were each placed again in the same corner of the apparatus in the trial session, and were allowed to locate and drink the water in the alcove. The elapsed times until the first entry into the alcove (entry latency, EL), until the initiation of drinking from the water tube (drinking latency, DL), and until the first touching/sniffing/licking of the water tube (contacting latency, CL) were measured.

### Primary Hippocampal Neuron (PHN) Culture and Treatments

Primary hippocampal neuron (PHN) samples were obtained from 1-day-old Sprague-Dawley rat pups. Cells were dissociated from newly dissected hippocampi with mechanical disruption in the presence of DNase and trypsin and then plated in poly-L-lysine-precoated six-well plates. Cells were seeded at a density of 2 × 10^6^ cells per well in Neurobasal^®^ Medium (1X) that was supplemented with 0.5 mM GlutaMAX^™^-I, B-27^®^ incubated at 37°C, 5% CO_2_. The medium was changed after 4 days. Then the cells were incubated with IGF-I (final concentration of 100 nM, PreProTech, Rocky Hill, NJ, USA) in the presence or absence of 50 μM ERK1/2 antagonist PD098059, 4 μM RSK antagonist BI-D1870, or 10 μM DA (Yang et al., 2006). Additionally, transfections of IGF-I siRNA/scrambled siRNA (Santa Cruz, CA, USA) into PHNs were performed with Lipofectamine 2000 (Invitrogen) according to the manufacturer’s protocol.

### Determination of DA Levels

A total of 300–800 ml of 0.4 M HClO_4_, which contained 0.1% (w/v) Na_2_S_2_O_5_, was added to the liver/serum/hippocampus sample. Then the mixture was homogenized by sonication (Labsonic-U-Braun). The homogenates were centrifuged at 200,009 g for 15 min at 4°C. Then aliquots of the supernatants were taken from analysis of DA using high-performance liquid chromatography (HPLC) with electrochemical detection using modifications in the mobile phase.

### Immunoprecipitation

Lysates were centrifuged, and the supernatants were then incubated with antibodies overnight at 4°C. They were subsequently incubated with protein G-agarose beads (Millipore) for 5 h at 4°C. Beads were washed three times with lysis buffer. Immunoprecipitated proteins were resolved by SDS-PAGE. Proteins were probed using primary and secondary antibodies following electroblotting. Blots were then analyzed using Quantity One (National Institutes of Health, Bethesda, MD, USA) and normalized to the respective loading controls. Data are expressed as fold changes relative to controls from three or four independent experiments that were performed independently.

### RT-PCR

Total RNA was isolated using a Qiagen RNA-Easy kit according to the manufacturer’s instructions. cDNA was created using oligo (dT), 0.1 M DTT, dNTP, RNaseOUT, Moloney murine leukemia virus reverse transcriptase, and 5× FS Buffer (all from Invitrogen). Amplification was carried out with PCR Master Mix (Promega). Amplified products were electrophoresed using 2% agarose gels, visualized after EtBr staining, and normalized to GAPDH. The following primers (Invitrogen) were used for murine genes: IGF-I: forward 5′-TCTGTGGAGAGCGAGGCTTT-3′ and reverse 5′-CACGTGACCGCCTTGCA-3′.

### Immunoblotting (IB)

PHNs or hippocampal tissues were harvested in lysis buffer (Sigma-Aldrich). The total protein was measured with a bicinchoninic acid protein assay (Amresco). Samples of 50 μg of protein were separated by SDS-PAGE and then were electroblotted to PVDF membranes. The membranes were blocked by incubation in 5% non-fat dry milk dissolved in TBS-T (150 mM NaCl, 0.05% Tween, and 2050 mM Tris). Proteins were probed using a primary antibody following electroblotting: pERK1/2 (ERK1 (pThr202/pTyr204) + ERK2 (pThr185/pTyr187)) (monoclonal/polyclonal, 1:1000), ERK1/2 (monoclonal/polyclonal, 1:1000), pnNOS Ser847 (monoclonal, 1:1000), pnNOS Ser1417 (monoclonal, 1:1000), nNOS (monoclonal, 1:2000), PSD95 (monoclonal, 1:2000), β-actin (monoclonal, 1:1000; Abcam), pRSK Ser369 (monoclonal, 1:1500; Biorbyt), or RSK (monoclonal, 1:5000; Biorbyt). Horseradish peroxidase-conjugated anti-rabbit secondary antibody (Abcam) was then used. Protein bands detected by antibodies were visualized by ECL reagent (Pierce) after extensive washing and were then exposed on Kodak BioMax film (Kodak). The films were scanned and the band intensities were quantified using Quantity One software. Densitometrical measurements were expressed as folds of proteins relative to GAPDH expression levels.

### Immunofluorescence (IF) Staining

If appropriate, for brain tissues, four-micron frozen brain sections that were fixed in 4% formaldehyde or acetone were blocked for endogenous peroxidase activity with 0.03% H_2_O_2_. PHNs were cultured on glass coverslips that were precoated with poly-L-lysine (Sigma-Aldrich) and then were fixed with 4% paraformaldehyde for 30 min and then treated with 0.1% Triton X-100 at room temperature for 10 min. Blocking was achieved with PBS that contained 5% normal goat serum at room temperature for 1 h.

Sections were then incubated at 4°C overnight with the following primary antibodies: IGF-I (monoclonal, 1:200), pERK1/2 (monoclonal, 1:400), pnNOS Ser1417 (monoclonal, 1:200), MAP2 (monoclonal, 1:500; Abcam), pRSK (monoclonal, 1:400; Biorbyt). Binding of primary antibodies was revealed by incubating the sections for 30 min with Alexa Fluor 488 (green)/Alexa Fluor 594 (red)-conjugated secondary antibodies (Abcam) or with horseradish peroxidase-labeled secondary antibodies (Abcam). They were then visualized by diaminobenzidine.

### Statistical Analysis

Data were analyzed by SPSS software (version 11.5; 2002) and are presented as mean ± SD. Statistical significance between groups was determined by a one-way analysis of variance (ANOVA) and parametric tests. Dunnett’s test was used for *post hoc* between-group comparisons whenever indicated by ANOVA. Student’s *t tests* for independent samples were used to analyze differences between two groups. Values of *P* < 0.01 or *P* < 0.05 were considered statistically significant.

## Results

### IGF-I Is Downregulated in MHE and DA-Treated Rats

We first tried to determine whether IGF-I had any antagonistic association with DA in the brains of MHE rats. RT-PCR showed that IGF-I transcription levels were lower in MHE rats (*F*_(1,23)_ = 6.3902, *p* < 0.05) and DA-treated rats (*F*_(1,18)_ = 6.443, *p* < 0.01) than in controls (Figure 1A). Immunoblotting (IB) revealed lower expression of IGF-I in MHE rats (*F*_(1,23)_ = 6.639, *p* < 0.05) and DA-treated rats (*F*_(1,18)_ = 6.846, *p* < 0.05) than in controls (Figures 1B,C). Double Immunofluorescence (IF) staining using anti-IGF-I antibodies and anti-MAP2 antibodies showed downregulation of IGF-I in MHE rats and DA-treated rats relative controls (Figure 1D).

**Figure 1:** Dopamine (DA) induces downregulation of Insulin-like growth factor I (IGF-I) in minimal hepatic encephalopathy (MHE) and DA-treated rats. **(A)** Assay for IGF-I mRNAs of hippocampal lysates from MHE rats (*n* = 13) or DA-treated rats (*n* = 10) by RT-PCR. **(B,C)** Immunoblot (IB) analysis of hippocampal lysates from MHE rats or DA-treated rats using anti-IGF-I and anti-β-actin antibodies and subsequent densitometry. **(D)** Double immunofluorescence (IF) staining of brain sections from MHE rats or DA-treated rats using antibodies against IGF-I (red) and mitogen-activated protein 2 (MAP2; green). **(E)** H&E staining of liver sections from MHE rats with IGF-I administration. Scale bar, 50 μm. **(F)** Sirius red staining of liver sections from MHE rats with IGF-I administration. Scale bar, 50 μm. Data are shown as mean ± SD. *P < 0.05. Scale bar, 25 μm. MRGD, merged image.

As shown in Figure 1E, regenerating hepatic nodules and inflammatory cell infiltration composed of lymphocytes and plasma cells were presented on HE staining in the liver of MHE rats, which were reversed by IGF-I administration. Likewise, by sirius red staining, fibrous septa formation was observed (Figure 1F) in the liver of MHE rats, which were also recovered to the normal level by IGF-I administration. These observations suggested that IGF-I had the ability to improve the liver cirrhosis.

### IGF-I Improves Memory Impairment in DA-Treated and MHE Rats

Given that IGF-I was reported to improve cognitive function (Arwert et al., 2005), we examined the effect of IGF-I on memory impairment in MHE. In the Y-maze test, the SA%, which was significantly higher in MHE (*F*_(2,37)_ = 4.3876, *p* < 0.05) and DA-treated (*F*_(2,27)_ = 4.764, *p* < 0.05) rats, returned to normal levels after IGF-I treatment (Figure 2A). In the water-finding task, the significant delay in CL, EL and DL detected in MHE (*F*_(2,37)_ = 4.777, *p* < 0.05) and DA-treated (*F*_(2,27)_ = 4.8354, *p* < 0.05) rats was ameliorated by IGF-I treatment (Figure 2B). These results indicated that DA impaired cognitive function by downregulating IGF-I in MHE rats.

**Figure 2:** IGF-I improves memory impairment in MHE and DA-treated rats. **(A)** Y-maze test of MHE rats (*n* = 13) or DA-treated rats (*n* = 10) with or without IGF-I administration (spontaneous alternation percentage, SA%). **(B)** Water-finding task of MHE rats or DA-treated rats with or without IGF-I administration (EL, entry latency; CL, contacting latency; DL, drinking latency). Data are shown as mean ± *SD*. *P < 0.05, **P < 0.01, ^#^*P* < 0.05.

### IGF-I Facilitated Inactivation of nNOS in PHNs

IGF-I contributes to the modulation of cognitive function (Broughton and Partridge, 2009), and PSD95 binds to nNOS to trigger nNOS enzyme activity, which causes neurotoxicity (Fukaya and Watanabe, 2000; Hu et al., 2013). Hence, we thought that IGF-I might prevent cognitive decline via disruption of the PSD95–nNOS interaction. We confirmed the PSD95–nNOS interaction by immunoprecipiton. Lysates from PHNs with IGF-I treatment were immunoprecipited with an anti-nNOS antibody. As predicted, IGF-I induced an increase in the amount of PSD95 that co-immunoprecipitated with nNOS (Figure 3A). Lysates were then immunoprecipitated with anti-PSD95 antibody, and, as predicted, IGF-I increased the amount of nNOS that coimmunoprecipitated with PSD95 (Figure 3B).

**Figure 3:** IGF-I triggers phosphorylation of neuronal nitric oxide synthase (nNOS) and destruction of postsynaptic density protein 95 (PSD95)–nNOS interaction in primary hippocampal neurons (PHNs). **(A)** Immunoprecipitation of lysates of PHNs with IGF-I treatment using control IgG or anti-/nNOS antibodies. Complexes were immunoblotted with anti-PSD95/nNOS antibodies. **(B)** Immunoprecipitation of lysates of PHNs with insulin treatment with control IgG or anti-PSD95 antibodies. Complexes were immunoblotted with anti-nNOS/PSD95 antibodies. **(C,D)** IB analysis of lysates of PHNs with IGF-I treatment using anti-pnNOS Ser1417/Ser847 and anti-nNOS antibodies and subsequent densitometry. **(E)** Double IF staining of PHNs with IGF-I treatment using antibodies against pnNOS Ser1417 (red) and MAP2 (green). **(F,G)** IB analysis of lysates of PHNs after IGF-I siRNA transfection using anti-pnNOS Ser1417/Ser847 and anti-nNOS antibodies and subsequent densitometry. Data are shown as mean ± SD. *P < 0.05, **P < 0.01. Scr, scramble. Scale bar, 25 μm. MRGD, merged image.

Phosphorylation of nNOS diminishes enzyme activity (Bredt et al., 1992) and protects the subject from neurotoxicity (Dawson et al., 1993). We therefore determined whether IGF-I stimulated the phosphorylation of nNOS and whether this disrupted the PSD95–nNOS interaction. IB showed that IGF-I stimulated nNOS phosphorylation at Ser847 and Ser1417 significantly more than in controls (Figures 3C,D). IF staining showed considerably more pnNOS Ser1417 expression in the IGF-I-treated PHNs than in controls (Figure 3E). We further assessed the effect of IGF-I on nNOS activity using IGF-I siRNA. IB for lysates from PHNs with knockdown of IGF-I revealed lower levels of pnNOS Ser847 and Ser1417 than in controls (Figures 3F,G). These data indicated that IGF-I disrupted the interaction of PSD95 with nNOS by phosphorylation of nNOS.

### IGF-I Promotes Activation of ERK1/2/RSK Signaling

RSK is known to be directly activated by ERK1/2 (Scimeca et al., 1992), so we further examined the mechanisms underlying of the effect of IGF-I on the relationship between nNOS and RSK via ERK1/2. IB showed cells treated with IGF-I had more phosphorylated RSK than controls (Figures 4A,B). IF staining also showed an IGF-I-induced increase in phosphorylated RSK in PHNs over control levels (Figure 4C). As shown in Figures 4D,E, IB analysis indicated that the amount of phosphorylated RSK was reduced by knockdown of IGF-I. IB from cell lysates showed that the phosphorylation of ERK1/2 became higher in cells exposed to IGF-I than in untreated controls (Figures 4F,G). IF staining indicated that IGF-I stimulated an increase in the number of pERK1/2-positive PHNs over control levels (Figure 4H). IB for lysates from PHNs with knockdown of IGF-I indicated a decrease in the phosphorylation of ERK1/2 relative to controls (Figures 4I,J). In summary, these results highlighted the important role of ERK1/2/RSK signaling in IGF-I signaling. Use of PD098059 abrogated IGF-I-stimulated an increase in pRSK over controls (Figures 4K,L).

**Figure 4:** IGF-I potentiates activation of extracellular signal-regulated kinase 1/2/ribosomal S6 protein kinase (ERK1/2/RSK) signaling. **(A,B)** IB analysis of lysates of PHNs with IGF-I treatment using anti-pRSK and anti-RSK antibodies and subsequent densitometry. **(C)** Double IF staining of PHNs with IGF-I treatment using antibodies against pRSK (red) and MAP2 (green). **(D,E)** IB analysis of lysates of PHNs after IGF-I siRNA transfection using anti-pRSK antibodies and subsequent densitometry. **(F,G)** IB analysis of lysates of PHNs with IGF-I treatment using anti- pERK1/2 and anti-ERK1/2 antibodies and subsequent densitometry. **(H)** Double IF staining of PHNs with IGF-I treatment using antibodies against pERK1/2 (red) and MAP2 (green). **(I,J)** IB analysis of lysates of PHNs after IGF-I siRNA transfection using anti-pERK1/2 antibodies and subsequent densitometry.** (K,L)** IB analysis of lysates of PHNs with IGF-I treatment in the absence or presence of PD098059 using anti-pRSK and anti-RSK antibodies and subsequent densitometry. Data are shown as mean ± SD. *P < 0.05, **P < 0.01. Scr, scramble. Scale bar, 25 mm. MRGD, merged image.

### IGF-I Triggers ERK1/2/RSK Axis to Disrupt PSD95–nNOS Interaction in PHNs

Next, we examined whether nNOS took part in the signaling cascade involved in IGF-I-induced stimulation of the ERK1/2-RSK pathway. Application of PD098059 abrogated the IGF-I-stimulated increase of pnNOS Ser1417 and Ser847 (Figures 5A,B). IB analysis showed that the addition of BI-D1870 reversed the increase in nNOS phosphorylation at Ser847 and Ser1417 in PHNs in response to IGF-I (Figures 5C,D).

**Figure 5:** IGF-I-induced phosphorylation of nNOS depends on ERK1/2/RSK signaling.** (A,B)** IB analysis of lysates of PHNs with or without IGF-I treatment in the absence or presence of PD098059 using anti-pnNOS Ser1417/Ser847 and anti-nNOS antibodies and subsequent densitometry. **(C,D)** IB analysis of lysates of PHNs with or without IGF-I treatment in the absence or presence of BI-D1870 using anti-pnNOS Ser1417/Ser847 and anti-nNOS antibodies and subsequent densitometry. Data are shown as mean ± SD. *P < 0.05.

We then confirmed the effect of the ERK1/2–RSK pathway on the nNOS–PSD95 interaction mediated by IGF-I. As determined by coimmunoprecipitation with an anti-nNOS antibody, IGF-I induced a decrease in PSD95, which coimmunoprecipitated with nNOS, and PD098059 abrogated the effect of IGF-I (Figure 6A). Coimmunoprecipitation with anti-PSD95 antibody revealed that, as predicted, IGF-I decreased the amount of nNOS that coimmunoprecipitated with pPSD95, and this decrease was eliminated by PD098059 (Figure 6B). Meanwhile, in coimmunoprecipitation with anti-nNOS antibody, IGF-I induced a decrease in the amount of PSD95 that coimmunoprecipitated with nNOS, and BI-D1870 abrogated this effect I (Figure 6C). In coimmunoprecipitation with anti-PSD95 antibody, as predicted, IGF-I decreased the amount of nNOS that coimmunoprecipitated with pPSD95, which was eliminated by BI-D1870 (Figure 6D). These data indicated that IGF-I-induced disruption of PSD95–nNOS interaction depends on the ERK1/2/RSK axis in PHNs.

**Figure 6:** IGF-I stimulates the disruption of RSK–nNOS interaction via ERK1/2/RSK signaling. **(A)** Immunoprecipitation of lysates of PHNs with or without IGF-I treatment in the absence or presence of PD098059 using control IgG or anti-nNOS antibodies. Complexes were immunoblotted with anti-nNOS/PSD95 antibodies.** (B)** Immunoprecipitation of lysates of PHNs with or without IGF-I treatment in the absence or presence of PD098059 using control IgG or anti-PSD95 antibodies. Complexes were immunoblotted with anti-PSD95/nNOS antibodies. **(C)** Immunoprecipitation of lysates of PHNs with or without IGF-I treatment in the absence or presence of BI-D1870 using control IgG or anti-nNOS antibodies. Complexes were immunoblotted with anti-nNOS/PSD95 antibodies.** (D)** Immunoprecipitation of lysates of PHNs with or without IGF-I treatment in the absence or presence of BI-D1870 using control IgG or anti-PSD95 antibodies. Complexes were immunoblotted with anti-PSD95/nNOS antibodies.

### IGF-I Disrupts DA-Induced PSD95–nNOS Interaction in PHNs

We found that DA impaired learning and memory in MHE rats in a previous study (Ding et al., 2013, 2014a,b,c). In this study, we assessed the effect of DA on the IGF-I-mediated ERK1/2/RSK pathway *in vitro*. RT-PCR showed that DA resulted in significantly lower IGF-I mRNA levels than in controls (Figure 7A). IB revealed decreased expression of IGF-I in PHNs with DA treatment compared to controls (Figures 7B,C). IF staining showed that the IGF-I levels were significantly lower in PHNs in response to DA than in controls (Figure 7D). IB analysis showed that the exposure of the PHNs to DA blocked the IGF-I-induced increase in expression of pRSK (Figures 7E,F). As shown in Figures 7G,H, IGF-I-stimulated elevation in the expression of ERK1/2 was eliminated by the addition of DA. In this way, DA was shown to impair IGF-I-mediated disruption of PSD95–nNOS interaction *in vitro*.

**Figure 7:** DA downregulated IGF-I to block the disruption of PSD95–nNOS interaction. **(A)** Assay for IGF-I mRNAs of lysates of PHNs with DA treatment for 6 h by RT-PCR. **(B,C)** IB analysis of lysates of PHNs with DA treatment using anti-IGF-I and anti-β-actin antibodies and subsequent densitometry. **(D)** Double IF staining of PHNs with DA treatment using antibodies against IGF-I (red) and MAP2 (green). **(E,F)** IB analysis of lysates of PHNs with or without IGF-I treatment in the absence or presence of DA using anti-pRSK and anti-RSK antibodies and subsequent densitometry. **(G,H)** IB analysis of lysates of PHNs with or without IGF-I treatment in the absence or presence of DA using anti-pERK1/2 and anti-ERK1/2 antibodies and subsequent densitometry. **(I)** Immunoprecipitation of lysates of PHNs with or without IGF-I treatment in the absence or presence of DA using control IgG and anti-nNOS antibodies. Complexes were immunoblotted with anti-PSD95/nNOS antibodies. **(J)** Immunoprecipitation of lysates of PHNs with or without IGF-I treatment in the absence or presence of DA using control IgG or anti-PSD95 antibodies. Complexes were immunoblotted with anti-PSD95/nNOS antibodies. Data are shown as mean ± SD. *P < 0.05, **P < 0.01. Scr, scramble. Scale bar, 25 μm. MRGD, merged image.

We determined the effect of DA on the IGF-I-mediated PSD95–nNOS interaction in PHNs. Immunoprecipitation with an anti-nNOS antibody showed that, as predicted, DA blocked the IGF-I-induced decrease in the amount of PSD95 that coimmunoprecipitated with nNOS (Figure 7I). Meanwhile, immunoprecipitation with anti-PSD95 antibody showed that IGF-I decreased the amount of nNOS that coimmunoprecipitated with PSD95, which was abrogated by DA (Figure 7J).

### IGF-I Inactivates ERK1/2/RSK Axis in MHE and DA-Treated Rats

Next, we checked whether the activity of the ERK1/2/RSK pathway seen in PHNs exposed to DA or IGF-I (Figure 7) was also present *in vivo*. As indicated by the IB analysis shown in Figures 8A,B, there was a decrease in the phosphorylation of RSK in the hippocampi of MHE rats and it was reversed with the administration of IGF-I (*F*_(2,37)_ = 4.345, *p* < 0.05); likewise, the expression of pRSK was reduced in the DA-treated group and returned to normal levels after the administration of IGF-I (Figures 8A,B; *F*_(2,27)_ = 4.509, *p* < 0.05). Similarly, IF staining confirmed that MHE rats given IGF-I displayed increased expression of pRSK, and administration of IGF-I to DA-treated rats also elevated expression of pRSK (Figure 8C). IB analysis showed decreased phosphorylation of ERK1/2 in MHE rats, and administration of IGF-I increased the phosphorylation of ERK1/2 (*F*_(2,37)_ = 4.468, *p* < 0.05). Decreased phosphorylation of ERK1/2 was also found in DA-treated rats and was reversed by administration of IGF-I (Figures 8D,E; *F*_(2,27)_ = 4.554, *p* < 0.05). Similarly, IF staining showed decreased pERK1/2 levels in MHE rats, and IGF-I induced a significant increase in pERK1/2 (Figure 8F). Pronounced pERK1/2 levels were significantly lower in DA-treated rats relative to controls. These levels were increased by the administration of IGF-I (Figure 8F). These results indicated that IGF-I reversed the DA-induced inactivation of the ERK1/2/RSK pathway in MHE.

**Figure 8:** IGF-I activates ERK1/2/RSK pathway in MHE and DA-treated rats. **(A,B)** IB analysis of hippocampal lysates of hippocampal lysates from MHE rats (*n* = 26) or DA-treated rats (*n* = 20) with or without IGF-I administration using anti-pRSK and anti-RSK antibodies and subsequent densitometry. **(C)** Double IF staining of brain sections from MHE rats or DA-treated rats with administration using antibodies against pRSK (red) and MAP2 (green). **(D,E)** IB analysis of hippocampal lysates from MHE rats or DA-treated rats with or without IGF-I administration using anti-pERK1/2 and anti-ERK1/2 antibodies and subsequent densitometry. **(F)** Double IF staining of brain sections from MHE rats or DA-treated rats with or without IGF-I administration using antibodies against pERK1/2 (red) and MAP2 (green). Data are shown as mean ± SD. *P < 0.05, **P < 0.01. Scale bar, 25 μm. MRGD, merged image.

### DA Induced Cognitive Loss via PSD95–nNOS Interaction in MHE Rats

We determined whether disruption of PSD95–nNOS interaction was involved in the cognitive decline in MHE. In the Y-maze test, SA%, which was significantly higher in MHE rats (Figure 9A) and DA-treated rats (Figure 9B), returned to normal levels in response to treatment with IC87201, an inhibitor of interference with the nNOS-PSD95 interaction (*F*_(2,37)_ = 4.489, *p* < 0.05). In the water-finding task, significant delays in CL, EL, and DL were measured in DA rats (Figure 9C) and MHE-treated rats (Figure 9D), the effect was ameliorated by IC87201 treatment (*F*_(2,37)_ = 4.318, *p* < 0.05). These results indicate that the PSD95–nNOS interaction was associated with pathogenesis of MHE.

**Figure 9:** DA triggers PSD95–nNOS interaction *in vivo*. **(A)** Y-maze test of MHE rats (*n* = 26) with or without IC87201 administration (SA%). **(B)** Y-maze test of DA-treated rats (*n* = 20) with or without IC87201 administration. **(C)** Water-finding task of MHE rats with or without IC87201 administration. **(D)** Water-finding task of DA-treated rats with or without IC87201 administration. Data are shown as mean ± SD. **P < 0.01.

### IGF-I Impairs Interaction of PSD95 and nNOS in MHE and DA-Treated Rats

We then determined whether the association of nNOS with PSD95 that was seen in PHNs exposed to DA or IGF-I (Figure 7) was also observable *in vivo*. We confirmed RSK–nNOS interactions *in vivo*. Lysates were then immunoprecipited with an anti-nNOS antibody. As predicted, the amount of PSD95 that coimmunoprecipitated with nNOS was increased in MHE rats, which was reversed by IGF-I; the same pattern was observed in DA-treated rats (Figure 10A). Lysates were then immunoprecipitated with an anti-PSD95 antibody, and, as predicted, the amount of nNOS that co-immunoprecipitated with PSD95 was amplified in MHE rats, which was reversed by IGF-I; the same pattern was found in DA-treated rats (Figure 10B). As indicated by the IF staining in Figure 10C,we found that the expression of pnNOS Ser847 was increased in the hippocampal neurons of MHE rats and increased by IGF-I administration. Meanwhile, the expression of pnNOS Ser847 showed significant increases in the hippocampal neurons of DA-treated rats, and administration of IGF-I abolished the effect of DA. IF staining indicated that the decreased expression of pnNOS Ser1417 in the hippocampal neurons of MHE rats was overturned by the administration of IGF-I. Decreased expression of pnNOS Ser1417 was observed in the hippocampal neurons of rats that were treated with DA, and IGF-I administration reversed the effect of DA (Figure 10D). These results indicate that IGF-I prevented the DA-induced interaction of PSD95 and nNOS in MHE.

**Figure 10:** IGF-I disrupts the interaction of PSD95 and nNOS in MHE and DA-treated rats.** (A)** Immunoprecipitation of lysates of MHE rats (*n* = 26) or DA-treated rats (*n* = 20) with or without IGF-I administration using control IgG and anti-nNOS antibodies. Complexes were immunoblotted with anti-PSD95/nNOS antibodies. **(B)** Immunoprecipitation of lysates of MHE rats or DA-treated rats with or without IGF-I administration using control IgG or anti-PSD95 antibodies. Complexes were immunoblotted with anti-nNOS/PSD95 antibodies. **(C)** Double IF staining of brain sections from MHE rats and DA-treated rats with or without administration using antibodies against pnNOS Ser847 (red) and MAP2 (green). **(D)** Double IF staining of brain sections from MHE rats and DA-treated rats with or without IGF-I administration using antibodies against pnNOS Ser1417 (red) and MAP2 (green). Scale bar, 25 μm. MRGD, merged image.

## Discussion

IGF-1, mainly synthesized by the liver, plays an important role in metabolism (Bonefeld and Møller, 2011). The liver cirrhosis in animal models and in patients was observed to be improved by the systemic administration of IGF-1 (Castilla-Cortazar et al., 1997; Conchillo et al., 2005; Sobrevals et al., 2010). Our results demonstrate that IGF-1 has endogenous defense mechanisms against liver cirrhosis in MHE and provide support for use of IGF-1 against cognitive decline and MHE pathology via an antifibrotic effect (Blaas et al., 2010).

Our results have significance in human pathology and provide support for use of IGF-I in MHE. It is demonstrated that IGF-I has a beneficial effect on liver cirrhosis in MHE (Blaas et al., 2010). Our results suggest that certain growth factors may have endogenous defense mechanisms against cognitive decline and MHE pathology via an antifibrotic effect. Most significantly, it means that IGF-I acts on both of liver and brain to overall ameliorate MHE.

Furthermore, studies have revealed that PSD95 interacts with nNOS to activate nNOS enzyme activity, leading to neurotoxicity (Fukaya and Watanabe, 2000; Hu et al., 2013). Thus, activated nNOS plays critical roles in MHE and PSD95. Our study showed that MHE is caused by the interaction between nNOS and PSD95. Therefore, dissociating this interaction blocks DA-induced MHE. IGF-I disrupts the interaction between nNOS and PSD95 to inhibit downstream nNOS signaling without blocking synaptic activity. This intervention was shown to be neuroprotective with a wider therapeutic window and fewer side effects.

Phosphorylation of nNOS is considered an important mechanism for the regulation of nNOS function. nNOS is phosphorylated at different residues by various protein kinases, and phosphorylation is considered to be a main mechanism that modulates nNOS function to decrease NO production. This study provided significant corroboration of the biological effects of nNOS phosphorylation, which could play a role in neuroprotection (Kasamatsu et al., 2014). Phosphorylation of nNOS results in diminished enzyme activity *in vitro* (Bredt et al., 1992) and further prevents neurotoxicity (Dawson et al., 1993). nNOS phosphorylation seems to be a key step in neuroprotection with the disruption of nNOS–PSD95 interactions. The net effect is that DA impedes the phosphorylation of nNOS by IGF-I, abrogating memory signaling. However, our results indicate that disruption of the nNOS–PSD95 complex should specifically be regulated by IGF-I is beneficial for memory function. The results showed that IGF-I markedly disrupted the PSD95–nNOS interaction and significantly inhibited the phosphorylation of nNOS without affecting the total nNOS expression level. This finding indicated that IGF-I triggers the phosphorylation of nNOS, which prevents the formation of the PSD95–nNOS complex and the activation of nNOS, thereby leading to an improvement in memory and learning in MHE. Also, we observed that IGF-I did not affect total nNOS expression, the deficiency of which has been shown to impair learning and memory (Kelley et al., 2009) and produce aggressive behavior (Nelson et al., 1995). This suggests that IGF-I may have fewer side effects as a potential drug for MHE. Several conclusions may be derived from our results. First, contrary modulation of nNOS activation by neuroprotective factors, such as IGF-I or DA determines the progression of MHE pathology in rats. Therefore, the imbalance that was observed between these regulatory factors in MHE most likely also drives human pathology. ERK1/2-RSK signaling activates the phosphorylation of nNOS to inhibit the nNOS-PSD95 complex in PHNs in response to IGF-I, and DA exerts a neurotoxic effect by abolishing the disruption of interaction between nNOS and PSD95 induced by IGF-I in neurons.

IGF-I promotes the *in vitro* and *in vivo* activation of the mitogen-activated protein kinase (MAPK) pathway, specifically ERK1/2 (Castillo et al., 2006). RSK1–4 originates from four independent genes. RSKs work at the distal end of the Ras/MAPK signaling pathway. They are directly activated and phosphorylated by ERK1/2 (Frodin and Gammeltoft, 1999). In the adult and embryonic brains of humans and mice, RSK is expressed predominantly in the hippocampus, neocortex and cerebellum, which have important roles in cognitive function and learning (Zeniou et al., 2002). Our observations pointing to inactivation of nNOS provide a robust rationale for the involvement in damage to the ERK1/2-RSK signaling pathway in MHE pathology, as DA induces the desensitization of the ERK1/2-RSK signaling pathway in MHE neurons. Collectively, these findings indicate that the dysregulated activity of ERK1/2-RSK signaling to nNOS in neurons contributes to disease load in MHE. IGF-I likely stimulates the ERK1/2-RSK axis to phosphorylate nNOS, and GF-I induces the phosphorylation of RSK through activation of ERK1/2. Although the mechanisms underlying a potential protective role of other growth factors in MHE requires further study, our results indicate that IGF-I is neuroprotective at least in part by triggering the disruption of nNOS–PSD95 interaction in neuron.

In neurons, RSK is directly activated by ERK1/2, and thus is involved in the core signaling cascade, which has been implicated in synaptic plasticity and memory (Davis and Laroche, 2006). It has been reported that RSK-1 phosphorylates nNOS, resulting in a reduction in its NO synthesis activity (Song et al., 2007; Zhou and Zhu, 2009). The net effect is that RSK interacts with nNOS and phosphorylation is increased. Therefore, the neuroprotective loop probably involves nNOS. Additionally, high levels of DA in MHE rats leads to reduced IGF-I levels. A corollary of this is that a decrease in IGF-I is an activator of MHE and can be considered as a postulated “second hit” required for memory impairment. Our results support a functional relationship between nNOS and RSK. However, RSK activity affected nNOS activation in neurons in response to IGF-I via phosphorylation of nNOS. Thus, DA was found to inhibit the activity of RSK and dissociate it from a complex with nNOS; subsequently, nNOS binds to PSD95. This PSD95–nNOS complex has a pivital role in mediating neuronal toxicity. We speculate that in MHE, the interaction of PSD95 and nNOS may produce deteriorating effects at least in part by triggering memory impairment in neurons.

We observed that the activation of nNOS by IGF-I is the cognitive arm in neurons that remains inactive in MHE due to a vicious cycle produced by high levels of DA. The observed imbalance between these regulatory factors seen in MHE rats is likely to drive human pathology. As ERK1/2-RSK signaling stimulates phosphorylation of nNOS to inhibit the nNOS-PSD95 complex in PHNs in response to IGF-I, furthermore, DA is neurotoxic, by eradicating the disruption of the interaction induced by IGF-I in neurons between nNOS and PSD95 (Figure 11). Indeed, the nNOS–PSD95 interaction is augmented in MHE. Its inhibition is enough to restore cognitive performance in MHE rats. Our data indicated that nNOS activity through the ERK1/2/RSK protein kinase cascade has a significant role in MHE. Our results elucidated an underlying protective mechanism by IGF-I on DA-induced interactions of PSD95 and nNOS. It is clear, however, that DA uncouples RSK from nNOS only in neurons stimulated with IGF-I.

**Figure 11:** Homeostasis of IGF-I-mediated cognitive signaling in neurons. **(A)** IGF-I initiates its effects through the activation of ERK1/2. Once activated, phosphorylated tyrosine residues on ERK1/2 recruit downstream RSK, which phosphorylates nNOS and disrupts the interaction of nNOS with PSD95, leading to trigger the learning and memory. **(B)** DA antagonizes the effect of the IGF-I signaling pathway.

## Author Contributions

SD: statistics, drafting and finalizing manuscript; JY, WZ, XW, YL and JH: performed experiments; CW: statistical analysis; QZ: manuscript draft.

## Conflict of Interest Statement

The authors declare that the research was conducted in the absence of any commercial or financial relationships that could be construed as a potential conflict of interest.
